# Influence of the Clinical Nursing Pathway on Nursing Outcomes and Complications of Cervical Carcinoma Patients Undergoing Chemotherapy via PICC

**DOI:** 10.1155/2022/4040033

**Published:** 2022-09-30

**Authors:** Hongxia Tang, Li Gao, Yahui Li

**Affiliations:** ^1^Medical Oncology, Shaanxi Provincial Cancer Hospital, Xi'an 710061, Shaanxi, China; ^2^Department of Gynecology and Oncology, Shaanxi Cancer Hospital, Xi'an 710061, Shaanxi, China

## Abstract

**Background:**

Cervical Carcinoma (CC) is the second most common cause of death in women, with most patients being diagnosed at an advanced stage. The conventional treatment for CC, with a long chemotherapy treatment cycle, is less than satisfactory and will cause serious damage to the patient's blood vessels.

**Objective:**

To analyze the impact of the clinical nursing pathway (CNP) on the incidence of complications and adverse prognosis in patients undergoing chemotherapy for CC via peripherally inserted central catheters (PICC).

**Materials and Methods:**

This study enrolled 157 CC patients who underwent PICC chemotherapy in the Shaanxi Provincial Cancer Hospital between March 2017 and April 2020 and assigned them between the two groups according to different nursing interventions. Ninety-three patients treated with CNP intervention were included in the research group (RG), and sixty-four cases treated with the routine nursing intervention were included in the control group (CG). The self-care ability and intervention satisfaction of patients were assessed using the self-care ability scale and the intervention satisfaction questionnaire, respectively, both developed by our hospital. The complication rate was observed in both cohorts, and the adverse prognosis of patients was statistically analyzed. Finally, an assessment was made on the patients' quality of life (QOL) using the quality of life questionnaire core 30 (QLQ-C30).

**Results:**

Higher scores of self-management information, catheter nursing ability, self-care compliance, and abnormal situation management were determined in RG after the nursing intervention. RG also outperformed CG in the overall incidence rates of complications and poor prognosis. Moreover, RG presented statistically higher nursing satisfaction and QLQ-C30 scores than CG after the nursing intervention.

**Conclusion:**

CNP has a significant nursing effect on patients with CC treated with PICC chemotherapy, which can not only reduce the incidence of postchemotherapy complications but also improve patient prognosis, satisfaction, and life quality, with the value for clinical promotion.

## 1. Introduction

Cervical carcinoma (CC), one of the major health issues in women, is the second most common cause of death among women [1]. According to statistics, the age-standardized mortality of cervical cancer is 3.39 per 100,000 women, ranking seventh among women in terms of cancer mortality [2]. CC usually spreads locally through direct tumor invasion, which invades laterally into the parametrium and distally into the upper vagina but rarely into the anterior and posterior part of the bladder or rectum [3]. Most CC patients do not present any symptoms in the early stage, instead, they are only found to be in the advanced stages at the time of initial diagnosis as the disease progresses [4]. Currently, the clinical treatment of CC is mostly centered on surgery or chemotherapy, the latter of which is primarily provided intravenously, with a long treatment cycle and substantial damage to patients' blood vessels due to chemotherapeutic toxicity [5]. Therefore, better treatment is urgently needed, which is of great significance to improve the survival and quality of life (QOL) of such patients.

PICC has a wide range of applications in clinical intravenous chemotherapy for tumor patients. However, long-term indwelling catheters will always cause complications such as catheter-related infection, catheter detachment, and damage during treatment, and even thrombosis in severe cases, posing a threat to patients' health [6, 7]. Besides, CC patients need long-time nursing due to a long treatment cycle, which is easy to cause various problems [8]. And during nursing, there may be operational errors and improper methods, resulting in venous inflammation and injury of the puncture site, which will seriously compromise the patients' treatment effect and quality of life (QOL) [9]. Therefore, looking for a reasonable nursing program can effectively reduce the adverse situation and improve curative efficacy. As a comprehensive and interdisciplinary clinical nursing model, the clinical nursing pathway (CNP) is an intervention with patients as the core that provides reasonable guidance and arrangement for their treatment, rehabilitation, and discharge [10]. And the examination items and treatment methods of patients under this intervention are accurately recorded and described since patient admission for treatment and intervention [11]. Patients can also clearly understand their own nursing goals through CNP, thereby improving their treatment initiative and compliance, forming self-care ability and awareness, and improving treatment efficacy [12]. For example, studies have shown that nursing intervention for patients with PICC intervention can reduce complications in the course of treatment and improve treatment effects [13].

At present, there are many studies on PICC chemotherapy for CC, but the impact of CNP on complications and poor prognosis is rarely reported. Accordingly, CC patients receiving PICC chemotherapy were given CNP intervention to investigate the improvement effect of this care model on complications, poor prognosis, and QOL, so as to develop a realistic nursing program for such a patient population.

## 2. Data and Methods

### 2.1. Study Participants and Recruitment Criteria

This research included 157 cases of CC with PICC chemotherapy in the Shaanxi Provincial Cancer Hospital between March 2017 and April 2020 and assigned them between the two groups based on different nursing interventions. CNP intervention was used in the research group (RG; *n* = 93), and routine nursing intervention was used in the control group (CG; *n* = 64). Inclusion criteria are as follows: (1) patients in both groups were diagnosed with CC by colposcopy, cervical smear cytology, and biopsy [14] before admission and received PICC chemotherapy and clinical nursing intervention in our hospital; (2) both cohorts of patients had complete clinical general data and were willing to accept relevant nursing and treatment, with expected life expectancy >6 months, no dependence on alcohol and drugs, and the ability to correctly understand and answer the relevant contents of relevant scales. Exclusion criteria are as follows: (1) those undergoing other treatments or who did not cooperate with this research were excluded, as well as withdrawals and loss to follow-ups.

### 2.2. Ethical Considerations

Ethical approval has been obtained from the Shaanxi Provincial Cancer Hospital. All patients who participated in this study fully understood the purpose of this study and signed the informed consent.

### 2.3. Nursing Models

Patients in CG were given routine nursing intervention. Upon patient admission, the nursing staff explained the nursing intervention knowledge in detail to patients and disseminated health propaganda. In addition, routine PICC catheterization management was performed to evaluate the patient's vascular condition. And according to the doctor's advice, education on related issues such as surgery, chemotherapy, and follow-up PICC catheter maintenance were carried out. The patient's vital signs were also tested.

Patients in RG were intervened by CNP: (1) Formulation of PICC chemotherapy regimen: a tailored chemotherapy regimen was formulated according to each patient's specific situation. Before that, blood vessels at the puncture site and the systemic coagulation function of the patient were evaluated. Subsequently, PICC chemotherapy-relative information, nursing process, and operation methods were popularized among patients and their families, and targeted psychological intervention was carried out. In addition, patients were guided to exercise and do abdominal breathing and urged to maintain good hygiene habits and daily routines. (2) Operation and comfort during catheterization: the nursing staff guided the patient to lie in an appropriate position, with the arm at the puncture site extended to 90°. The nursing staff kindly inquired about the patient's feelings during the puncture. When the catheter was inserted 10–15 cm, the patient was instructed to tilt the head toward the puncturing end. Local compression and bandaging were carried out within 30 min postoperatively. In addition, the patient was told that the elbow with catheter placement should not bend within 24 hours, and a soft pillow was placed under the arm. The PICC catheterization record sheet was filled out in detail. The nursing staff was assigned to inspect the catheterization of patients within 12 hours of effective catheterization to avoid adverse reactions such as discomfort, phlebitis, and limb pain. (3) On the first day after catheter placement, the nursing staff was arranged to remove and change the dressing for the patient. After the bottom-up removal, the puncture site of the patient was carefully observed to record any abnormality. After that, the dressing of PICC was changed, and infusion connectors were replaced. The nursing staff was also there for regular maintenance and management. In addition, a 10 mL heparin solution was administered with a syringe for pulse flushing and positive pressure sealing before and after blood transfusion, drug administration, and infusion. (4) Recovery guidance was also provided for patients 2 to 6 days after catheterization, including hand movements such as forearm internal and external rotation. (5) On the seventh day of catheterization, the nursing staff replaced the application for the patient in time and told the patient to keep it dry to avoid dampness or pollution. (6) When the patient was about to be discharged from the hospital, the nursing staff taught the patient and their family the ways for catheter maintenance and listed the daily precautions after discharge. Regular phone calls were also made to visit the patient's recovery after discharge.

### 2.4. Clinical Outcomes

1. *Self-Management Ability*. Patients were scored for their self-care ability using the self-developedself-care ability scale for PICC chemotherapy from the following four items (each with a full score of 100 points): self-management information, catheter nursing ability, self-care compliance, and abnormal situation management. The higher the score after evaluation and statistics, the higher the patients' self-efficacy.
2. *Complications*. The incidence rates of catheter blockage, catheter detachment, infection, venous thrombosis, puncture site bleeding, and pressure ulcers during the nursing intervention were observed and recorded.
3. *Incidence of Adverse Prognosis*. The incidence of adverse prognosis after the nursing intervention was also observed and recorded.
4. *Nursing Satisfaction*. We scored patient satisfaction with the nursing service using the satisfaction questionnaire (score range: 0–100) developed by our hospital. Higher scores indicated higher patient satisfaction.
5. *QOL Questionnaire*. the quality of life questionnaire core 30 (QLQ-C30) (QLQ-C30) [15], assessed from 5 dimensions with a total score of 100 points for each, was utilized to assess patients' QOL. The score after the evaluation was positively associated with the QOL of patients.

### 2.5. Statistical Data Analysis

The collected data were statistically analyzed and visualized into figures using SPSS 21.0 (SPSS, Inc, Chicago, IL, USA) and GraphPad Prism 6.0 (GraphPad Software Inc., San Diego, CA, USA), respectively. The chi-square test or the continuity correction chi-square test (applied when the theoretical frequency of the chi-square test was less than 5) were used for inter-group comparisons of categorical data (smoking history, drinking history, etc.) and recorded as the number of cases/percentage (n (%)). Mean ± standard deviation (mean ± SD) was used to indicate the quantitative data such as average age and average course of disease; the differences between and within groups were identified by independent samples *t*-test and paired *t-test*, respectively. The threshold of significance was *P* < 0.05.

## 3. Results

### 3.1. Patient's Demographic Data

RG and CG showed no statistical significance in average age, average course of disease, body mass index, smoking history, drinking history, hypertension history, pathological stage, and other general clinical baseline data (*P* > 0.05) (Table 1).

### 3.2. Comparison of Self-Care Ability after Nursing Intervention

RG showed statistically higher scores in self-management information, catheter maintenance ability, self-care compliance, and abnormal situation management than CG after nursing intervention (*P* < 0.05) (Table 2).

### 3.3. Comparison of Complications after Nursing Intervention

The overall complication rate after the nursing intervention was 4.30% in RG and 18.75% in CG, with statistical significance (*P* < 0.05) (Table 3).

### 3.4. Analysis of Adverse Prognosis after Nursing Intervention

The incidence of adverse prognosis in RG after nursing intervention was 3.23%, significantly lower than that of 12.50% in CG (*P* < 0.05) (Table 4).

### 3.5. Comparison of Nursing Satisfaction

The statistics on nursing satisfaction revealed statistically higher scores of service timeliness, management standardization, service attitude, hospitalization environment, and comprehensive quality of nursing staff in RG compared with CG after nursing intervention (*P* < 0.05) (Figure 1).

### 3.6. Comparison of QLQ-C30 Scores before and after Nursing Intervention

We evaluated the scores of somatic, role, cognitive, emotional, and social functions of patients. After the intervention, the scores of all dimensions were found to be higher in RG compared with CG (*P* < 0.05) (Figure 2).

## 4. Discussion

CC is a common gynecological malignancy usually treated with surgery or radiotherapy/chemotherapy [16, 17]. The PICC catheterization provides a more effective infusion strategy for treatment, which decreases the damage caused by chemotherapeutics and repetitive arterial puncture [18]. However, most elderly patients with CC need catheter maintenance during inpatient chemotherapy, requiring guidance from professional medical staff to prevent complications and other adverse events during treatment that affect the overall treatment; hence, finding better nursing methods is critical [19].

In this study, we employed CNP to intervene in the self-care abilities, complications, adverse prognosis, and QOL of patients with CC receiving PICC chemotherapy. Patients' symptoms were found to be improved after CNP intervention. As indicated by Leung et al. [20], most patients cannot maintain PICC timely and correctly due to their low educational cognition and a lack of awareness of the importance of regular PICC maintenance. Hence, it is very important to give nursing intervention during PICC treatment. In this study, targeted knowledge popularization of PICC and catheter maintenance guidance was carried out for patients to improve their treatment compliance. Unsurprisingly, statistically higher scores of self-management information, catheter nursing ability, self-care compliance, and abnormal situation management were determined in RG after the nursing intervention. It shows that CNP intervention can actively provide professional health guidance for patients from multiple angles, fully mobilize patients' self-care ability, and consciousness in the intervention process and effectively improve their self-management ability, all of which contribute to health maintenance. However, it is shown that although PICC is the main venous access for cancer patients receiving chemotherapy and nutritional support, the resulting venous thrombosis is also one of the most common complications [21].

Wang et al. [22] reported that nursing intervention for patients with malignant hematological diseases treated by PICC could effectively reduce PICC-induced bloodstream infection and thrombosis. In this study, RG exhibited an obviously lower complication rate and a lower adverse prognosis rate. This shows that the popularization of PICC catheterization related knowledge for patients can help prevent catheter blockage, catheter detachment, venous thrombosis, and other adverse events. It can also increase patients' knowledge of the efficacy of self-treatment, minimizing complications, and poor prognosis. In the study of Xiao et al. [23] on cerebral infarction, it was suggested that the application of CNP can reduce complications and recurrence, which is consistent with our study.

Research shows that traditional nursing approaches lack goals, systems, and plans, which reduce therapeutic efficacy [24]. CNP, on the other hand, can establish appropriate plans based on the patients' conditions, execute targeted nursing measures, and increase patients' awareness of their problems and treatments, all of which can help improve the therapeutic effect [25]. In this study, patients were invited to score their satisfaction with the nursing care they received, and unsurprisingly, a higher satisfaction score was determined in RG. It shows that patients have high recognition and good feedback on this nursing, providing a powerful reference for subsequent clinical application. As we all know, CC can significantly affect the QOL of patients, so efforts should be made to improve patients' life quality [26]. In this paper, the QLQ-C30 scores were statistically higher in RG after nursing. This may be due to the application of CNP intervention, which improves patients' cognition of PICC catheterization, reduces the incidence of complications during intervention and facilitates rehabilitation in various aspects, thus improving the QOL of patients. This is also consistent with the study of Liao et al. [27], who reported improved QOL of patients with hypertension and cerebral infarction by CNP.

## 5. Conclusion

In summary, for CC patients receiving PICC chemotherapy, CNP can significantly enhance their self-care ability and mitigate negative effects after PICC chemotherapy and improve their QOL and satisfaction with this nursing experience.

## Figures and Tables

**Figure 1:** Comparison of nursing satisfaction between the two groups of patients. (a) Service timeliness scores of both groups after nursing intervention. (b) Management standardization scores of both groups after nursing intervention. (c) Service attitude scores of both groups after nursing intervention. (d) Hospitalization environment scores of both groups after nursing intervention. (e) Comprehensive quality of nursing staff scores after nursing intervention in both groups. Note: ^*∗*^*P* < 0.05 between the two groups.

**Figure 2:** Comparison of QLQ-C30 scores between the two groups before and after the nursing intervention. (a) Somatic function scores of both groups after nursing intervention. (b) Role function scores of both groups after nursing intervention. (c) Cognitive function scores of both groups after nursing intervention. (d) Emotional function scores of both groups after nursing intervention. (e) Social function scores of both groups after nursing intervention. Note: ^*∗*^*P* < 0.05 between the two groups.

**Table 1:** Comparison of general data between the two groups (*n* (%) (mean ± SD).

Categories	Research group (*n* = 93)	Control group (*n* = 64)	t/*χ*^2^	*P*
Average age (years)	51.17 ± 5.62	49.59 ± 5.24	1.779	0.077

Average course of disease (years)	2.62 ± 0.96	2.97 ± 1.88	1.530	0.128

Body mass index (kg/m^2^)	23.68 ± 2.56	24.23 ± 3.98	1.054	0.294

Smoking history			1.553	0.216
Yes	33 (35.48)	29 (45.31)		
No	60 (64.52)	35 (54.69)		

Drinking history			0.179	0.672
Yes	38 (40.86)	24 (37.50)		
No	55 (59.14)	40 (62.50)		

History of hypertension			0.055	0.813
With	41 (44.09)	27 (42.19)		
Without	52 (55.91)	37 (57.81)		

TNM stage			1.061	0.303
I	35 (37.63)	19 (29.69)		
II	58 (62.37)	45 (70.31)		

**Table 2:** Comparison of self-management ability between the two groups after nursing (mean ± SD).

Groups	*n*	Self-managementinformation	Catheter maintenance ability	Self-care compliance	Abnormal situation management
Research group	93	91.43 ± 4.59	89.96 ± 6.31	94.16 ± 5.86	90.60 ± 7.55
Control group	64	83.50 ± 4.44	83.03 ± 4.78	81.45 ± 7.51	79.52 ± 6.51
*t value*	—	10.779	7.437	11.892	9.547
*P value*	—	<0.001	<0.001	<0.001	<0.001

**Table 3:** Comparison of complications after nursing intervention between the two groups (*n* (%)).

Categories	Research group (*n* = 93)	Control group (*n* = 64)	*χ* ^2^ value	*P* value
Catheter blockage	0 (0.00)	2 (3.13)	2.944	0.086
Catheter detachment	2 (2.15)	3 (4.69)	0.791	0.374
Infection	0 (0.00)	1 (1.56)	1.462	0.226
Venous thrombosis	0 (0.00)	1 (1.56)	1.462	0.226
Bleeding at puncture site	1 (1.08)	2 (3.13)	0.849	0.356
Pressure sores	1 (1.08)	3 (4.69)	1.992	0.158
Overall incidence	4 (4.30)	12 (18.75)	8.648	0.003

**Table 4:** Analysis of poor prognosis of patients in two groups after nursing intervention (*n* (%)).

Groups	*n*	Recurrence	Metastasis	Death	The total incidence of poor prognosis (%)
Research group	93	2 (2.15)	0 (0.00)	1 (1.08)	3 (3.23)
Control group	64	3 (4.69)	2 (3.13)	3 (4.69)	8 (12.50)
*t value*	—	0.791	2.944	1.992	5.005
*P value*	—	0.374	0.086	0.158	0.025

## Data Availability

The dataset used to support the findings of this study is available from the corresponding author upon request.
